The article "Stably Luminescent Staphylococcus aureus Clinical Strains for Use in Bioluminescent Imaging" was published in 2013. Journal: PLoS One.

# Stably Luminescent *Staphylococcus aureus* Clinical Strains for Use in Bioluminescent Imaging

**DOI:** 10.1371/journal.pone.0059232

**Published:** 2013-03-12

**Authors:** Roger D. Plaut, Christopher P. Mocca, Ranjani Prabhakara, Tod J. Merkel, Scott Stibitz

**Affiliations:** Division of Bacterial, Parasitic, and Allergenic Products, Center for Biologics Evaluation and Research, Food and Drug Administration, Bethesda, Maryland, United States of America; Universitätsklinikum Hamburg-Eppendorf, Germany

## Abstract

*In vivo* bioluminescent imaging permits the visualization of bacteria in live animals, allowing researchers to monitor, both temporally and spatially, the progression of infection in each animal. We sought to engineer stably luminescent clinical strains of *Staphylococcus aureus*, with the goal of using such strains in mouse models. The gram-positive shuttle vector pMAD was used as the backbone for an integration plasmid. A chloramphenicol resistance gene, a modified lux operon from *Photorhabdus luminescens*, and approximately 650 bp of homology to the chromosome of the USA300 *S. aureus* strain NRS384 were added, generating plasmid pRP1195. Electroporation into strain RN4220 followed by temperature shift led to integration of pRP1195 into the chromosome. The integrated plasmid was transferred to clinical strains by phage transduction. Luminescent strains displayed no *in vitro* growth defects. Moreover, luminescence was stable *in vitro* after three rounds of subculture over 48 hours of growth in the absence of antibiotics. Mice were infected with a luminescent strain of NRS384 in skin and intravenous models. In a mouse skin model, luminescent bacteria were present in lesions that formed and cleared over the course of several days, and in an intravenous model, bacteria inoculated in the mouse tail vein were observed spreading to multiple tissues. No statistically significant difference in virulence was observed between NRS384 and the luminescent strain in either infection model. These preliminary data suggest that this luminescent USA300 strain is suitable for use in mouse models. Similar strains were engineered using other sequenced clinical strains. Because these strains are stably luminescent, they should prove useful in animal models of infection.

## Introduction

*Staphylococcus aureus* is responsible for a variety of illnesses, including skin and soft tissue infections, pneumonia, septic arthritis, endocarditis, and osteomyelitis. The incidence of infections with antibiotic-resistant strains is increasing, with community-acquired methicillin-resistant *S. aureus* (CA-MRSA) becoming a particular concern (reviewed in [1]). Studies of these infections using animal models are facilitated by the use of bioluminescent imaging (BLI), which allows tracking of the spatial progression of infection in individual animals over time.

For use in BLI, bacterial strains should be clinically relevant and brightly and stably luminescent. Although there are several reports using luminescent *S. aureus* strains *in vivo* [2], [3], [4], [5], [6], the strains used are often not stably luminescent. One issue is that if the genes required for luminescence are carried on a plasmid, then the signal may be lost *in vivo* in the absence of antibiotic selection, due to plasmid segregation. Moreover, in some of these reports, the strains used in BLI were luminescent versions of laboratory-passaged strains, which may not be clinically relevant to current human diseases.

In this report, we describe an integrative plasmid developed to engineer stably and brightly luminescent clinical strains of *S. aureus*. In preliminary experiments, we used one of these strains, a luminescent version of the USA300 MRSA strain NRS384, in two mouse models of infection. We found that the luminescent strain was as virulent as the wild-type strain, and that progression of the infections could be followed easily over time using BLI. The integrative plasmid and the luminescent clinical strains described here should prove useful in these and other animal models of *S. aureus* infection.

## Materials and Methods

### Bacterial strains and plasmids

Bacterial strains and plasmids are listed in Table 1. The backbone for the integrative plasmid was the shuttle plasmid pMAD [7]. The kanamycin resistance gene *aphA(3)*, originally from *S. aureus* [8], was amplified from pSS4332 [9] and inserted at the BglII site of pMAD, yielding plasmid pRP1179. Approximately 660 bp in the area of USA300HOU_1102 (annotated as a pseudogene in the sequenced USA300 strain TCH1516 [10]) was amplified from the *S. aureus* USA300 strain NRS384 and inserted into BamHI/SalI-digested pRP1179, generating pRP1186. Next, a modified *luxBADCE* operon, originally from *Photorhabdus luminescens* [11], was amplified from a derivative of pSS4530 [12] such that the operon was under the control of a modified *gapA* promoter with consensus -35, extended -10, and -10 regions (TTGACA CTGCGTAAGGTTTGTGTTATAAT ) and inserted at the EagI site of pRP1186, yielding pRP1190. Separately, the chloramphenicol resistance gene *cat* (originally from pC194 [13]) was amplified from pBT2 [14], digested with KpnI, and inserted into similarly digested pMAD, generating plasmid pRP1192. Finally, a 6.8 kb BamHI-SalI fragment of pRP1190 (including the USA300HOU_1102 homology and the *lux* operon) was ligated with similarly digested pRP1192, generating pRP1195 (Fig. 1). Thus, pRP1190 (with *aphA(3)*) is suitable for use in *S. aureus* strains that are kanamycin-sensitive, whereas pRP1195 (with *cat*) is suitable for use in strains that are chloramphenicol-sensitive. Plasmids were transformed into RN4220 by electroporation as previously described [15] followed by growth at 30°C. For integration into the bacterial chromosome, strains were grown at 30°C overnight in tryptic soy broth (TSB) with 10 µg/ml chloramphenicol, followed by subculture (1∶100 dilution) in TSB without antibiotics at 30°C for 1–2 h, shift to 43°C for 6–7 h, serial dilution, plating on tryptic soy agar (TSA) with 10 µg/ml chloramphenicol, and overnight incubation at 43°C. Plates were imaged, and luminescent colonies were selected for further passage and analysis. Integration at the intended site was confirmed by PCR. Freely replicating or integrated plasmids were transferred to clinical strains by phi80 phage transduction as previously described [16].

**Figure 1:** Map of integrative plasmid pRP1195. Features added to the pMAD backbone as described in Materials and Methods include: *cm*, chloramphenicol resistance gene; homology, PCR fragment in the area of pseudogene USA300_HOU1102 amplified from NRS384; LuxB, A, D, C, and E, modified *lux* operon from *Photorhabdus luminescens*.

**Table 1:** Plasmids and strains used in this work.

Plasmid/strain	Description/features	Source/reference
Plasmids		
pMAD	*S. aureus* shuttle vector	[7]
pSS4530	modified *luxBADCE* operon	[11], [12]
pSS4332	source of kanamycin resistance gene *aphA(3)*	[8], [9]
pBT2	source of chloramphenicol resistance gene *cat*	[13], [14]
pRP1179	pMAD with *aphA(3)* from pSS4332	This work
pRP1186	pRP1179 with homology to USA300HOU_1102	This work
pRP1190	pRP1186 with *luxBADCE* from pSS4530, under control of modified *gapA* promoter	This work
pRP1192	pMAD with *cat* from pBT2	This work
pRP1195	pRP1192 with *luxBADCE* and homology to USA300HOU_1102 from pRP1190	This work
*S. aureus*		
RN4220	Restriction-deficient laboratory strain	[18]
NRS384	USA300-0114 CA-MRSA	NARSA collection
MW2	CA-MRSA	[19], [20]
Newman	Methicillin-sensitive	[21], [22]
SAP140	RN4220 with freely replicating pRP1195	This work
SAP143	RN4220 with pRP1195 integrated at USA300HOU_1102 (temperature shift of SAP140)	This work
SAP149	NRS384 with integrated pRP1195 via transduction from SAP143	This work
SAP224	NRS384 with freely replicating pRP1195 via transduction from SAP140	This work
SAP231	NRS384 with integrated pRP1195 (temperature shift of SAP224)	This work
SAP221	MW2 with freely replicating pRP1195 via transduction from SAP140	This work
SAP227	MW2 with integrated pRP1195 (temperature shift of SAP221)	This work
SAP217	Newman with freely replicating pRP1195 via transduction from SAP140	This work
SAP229	Newman with integrated pRP1195 (temperature shift of SAP217)	This work

### *In vitro* growth and luminescence

To assess the kinetics of growth *in vitro*, strains were grown overnight in TSB and subcultured at a dilution of 1∶100, and OD_600_ readings were taken at regular intervals. To assess the stability of luminescence following extended *in vitro* growth, strains were grown in TSB and subcultured three times (at 16, 24, and 40 h) in the absence of antibiotics, and after 48 h, serial dilutions were plated on TSA and incubated at 37°C.

### Mouse infections

Animal studies were conducted at the animal facility of the Center for Biologics Evaluation and Research, under the guidelines of the Institutional Animal Care and Use Committee (IACUC), which approved the animal protocols used. All efforts were undertaken to minimize animal suffering. For a skin and soft tissue model of infection, TSB without (NRS384) or with (SAP149) 10 µg/ml chloramphenicol was inoculated at a dilution of 1∶50 with an overnight culture, incubated at 37°C with shaking, grown to an OD_600_ of approximately 0.8, and then centrifuged at 4000× g for 15 min. The pellet was resuspended in PBS, and bacteria were counted using a hemocytometer and diluted in PBS to a concentration of 1.0×10^11^ cells/ml. The bacterial count was confirmed by serial dilution and plating of the suspension. BALB/c mice were anesthetized intraperitoneally with 2 mg ketamine (Ketaject, Phoenix Pharmaceutical, St. Joseph, MO) and 0.1 mg xylazine (AnaSed, Akorn, Decatur, IL). Left ears were swabbed with 70% isopropanol, and a Morrow Brown needle (Morrow Brown Allergy Diagnostics, Oakhurst, NJ) was used to administer 1.0×10^9^ CFU to the left ear of each mouse. The mean delivered dose was found to be approximately 2.0×10^7^ CFU/lesion with a standard deviation of 1.0×10^7^ CFU/lesion. Mice were euthanized on days 1, 4, and 7 following infection, and the left ears were cleansed with 70% ethanol. Ear pinnae were removed using sterile scissors and homogenized in 500 μl of PBS with a Polytron PT 1200 handheld homogenizer (Kinematica, Bohemia, NY). Serial dilutions were plated on TSA and incubated overnight at 37°C, and CFU per ml of homogenate was calculated.

For an intravenous model, TSB without (NRS384) or with (SAP149) 10 µg/ml chloramphenicol was inoculated at a dilution of 1∶100 with an overnight culture, incubated at 37°C with shaking, and grown to an OD_600_ of approximately 0.63. This absorbance reading was found to correspond to approximately 3.66×10^8^ CFU/ml (data not shown). The culture was centrifuged at 4000× g for 10 min, and the pellet was resuspended in PBS. BALB/c mice were injected via the tail vein with 2×10^7^ CFU of NRS384 or SAP149 in a volume of 100 µl. The dose was verified by serial dilution and plating on TSA. Over the course of 21 days, moribund mice were euthanized according to an IACUC-approved protocol.

### Imaging, image processing, and statistical analyses

To follow the progression of the infection, mice were imaged with an IVIS-50 instrument (Caliper Life Sciences, Hopkinton, MA) as previously described [12]. Agar plates were imaged with an LAS-3000 imaging system (Fujifilm Medical Systems, Stamford, CT). Typical settings for assessing luminescence were f/0.85, 1 min, no filter. Images were adjusted for brightness and contrast using PhotoShop CS3 (Adobe Systems, San Jose, CA). Prism 5 (GraphPad Software, La Jolla, CA) was used for statistical analyses.

## Results

### Development and integration of a luminescence plasmid

In order to engineer strains of *S. aureus* that would be stably luminescent, we sought to integrate a plasmid into the bacterial chromosome. The shuttle plasmid pMAD [7], which contains a temperature-sensitive replication module, was used as the backbone. Because some clinical strains already carry erythromycin resistance, a gene encoding resistance to chloramphenicol [13] was added. In a search for potential integration sites, we considered pseudogenes in the chromosome of the sequenced USA300 strain TCH1516 [10] (Accession NC_010079.1). We selected pseudogene USA300HOU_1102 (Gene ID: 5776586) as the site for integration, for the following reasons: 1) it is a pseudogene in several sequenced strains, decreasing the likelihood that insertion at that site would affect fitness or virulence; 2) flanking genes are encoded “toward” it, decreasing the likelihood of polar effects; and 3) the region is 98–100% conserved in 32 sequenced *S. aureus* strains, including strains commonly used in research (e.g., MW2, Newman, COL, and N315), enabling the use of homology cloned from one strain for integration of the plasmid into the chromosomes of multiple strains. A 662-bp PCR fragment in the area of pseudogene USA300HOU_1102 (coordinates 1171718-1172379) was amplified from the USA300 strain NRS384 and inserted into the plasmid, to permit integration of the plasmid into the bacterial chromosome via homologous recombination. Lastly, a modified *lux* operon originally from *Photorhabdus luminescens* [11], [12] was added, under the control of a strong constitutive promoter, leading to the development of the integrative plasmid pRP1195 (Fig. 1).

The plasmid was transformed by electroporation into the restriction-deficient laboratory strain RN4220, and chromosomal integrants were selected by temperature shift in the presence of chloramphenicol. Phage phi80 was used to transduce the integrated plasmid into the strains NRS384, MW2, and Newman. In later experiments, freely replicating plasmid pRP1195 was transduced into the clinical strains and then integrated into the chromosomes of those strains by temperature shift in the presence of chloramphenicol. The site of integration was confirmed by PCR (Fig. 2) and sequencing.

**Figure 2:** PCR analysis of plasmid integration. Primers specific for pRP1195 and chromosomal sequences were used in PCR reactions with chromosomal DNA from SAP231 (integrant) and NRS384 (WT) as templates. Primers used were: C1, (GCATGCCATTTTCTTTATCATAAGTG); C2, (CAGTTATGGTGGTCTTATAGAGAGAC); P1, (CAGTCAGAGGAGCGCCGACAACACC); P2, (TTTCGTTTGTTGAACTAATGGGTGC). Molecular weight in kilobases is indicated on the left.

### Evaluation of luminescent strains *in vitro*

The luminescent strains exhibited similar growth kinetics *in vitro*, relative to each other and to the parental strains (Fig. 3A). In order to assess the stability of the luminescence, the strains were grown in broth culture and subcultured three times over the course of 48 h in the absence of antibiotics, and serial dilutions were plated. All colonies were found to be luminescent (Fig. 3B), confirming the stability of the integrated plasmid *in vitro*.

**Figure 3:** Analysis of *in vitro* growth. A) *In vitro* growth curves. Strains were grown overnight in TSB with (luminescent strains) or without (parental strains) 10 µg/ml chloramphenicol and subcultured at a dilution of 1∶100 in TSB without antibiotic. MW2-Lux, SAP227; Newman-Lux, SAP229; NRS384-Lux, SAP231. B) Luminescence after *in vitro* outgrowth. SAP231 was grown in TSB and subcultured three times over the course of 48 h. Serial dilutions were plated on TSA in the absence of antibiotics, and plates were imaged as described in Materials and Methods.

### Animal infections

In an intravenous model, mice were injected via the tail vein with the wild-type USA300 strain (NRS384) or with the luminescent derivative (SAP149). When mice infected with the luminescent strain were imaged over the course of 6d, luminescent bacteria were apparent by day 1 and were observed to have spread throughout the body of each animal (Fig. 4A). Mice injected with either strain succumbed to the infection, with time of death varying from 1 to 21 days (Fig. 4B). There was no statistically significant difference between the survival curves of mice infected with each strain.

**Figure 4:** BALB/c intravenous infection with wild-type or luminescent NRS384. In an intravenous model, mice were injected via the tail vein with either the wild-type USA300 strain (NRS384) or the luminescent strain (SAP149). Mice injected with the luminescent strain were imaged over the course of 6d (A); images are representative. There was no statistically significant difference in survival of mice injected with the two strains (B) by either the log-rank (Mantel-Cox) Test (*P* = 0.46) or the Gehan-Breslow-Wilcoxon Test (*P* = 0.68); n = 20 mice per group.

In a skin and soft tissue model of infection, wild-type or luminescent bacteria were transferred to a Morrow-Brown needle and inoculated onto the left ear of mice. Mice infected with the luminescent strain SAP149 were imaged over the course of several days (Fig. 5A). Luminescence was apparent on day 1 following infection, increased over the course of 3–5 days, and then began to wane. By day 7, the infection had nearly cleared, as evidenced by the reduction in luminescence and confirmed by bacterial counts (Fig. 5B). There was no statistically significant difference in CFU per ml of ear pinna homogenate between mice infected with the luminescent strain and those infected with the wild-type USA300 strain, suggesting that integration of the plasmid into the bacterial chromosome did not affect virulence.

**Figure 5:** BALB/c skin and soft tissue infection with wild-type or luminescent NRS384. In a skin and soft tissue model (SSTI), mice were inoculated in the left ear with NRS384 or SAP149. Mice inoculated with SAP149 were imaged over the course of several days (A); images are representative. On days 1, 4, and 7 post infection, mice were euthanized and ear pinna homogenates were serially diluted and plated (B). There was no statistically significant difference in CFU recovered per ml of homogenate between mice infected with each strain (two-tailed t-test; *P* = 0.55; bars represent 95% confidence interval; n = 8 mice per group).

## Conclusions

In a previous study, we found that *Bacillus anthracis* engineered to be luminescent via integration of a plasmid by homologous recombination is very stably luminescent, even in the absence of antibiotic selection [12]. In the present work, we used a similar approach to engineer luminescent *S. aureus* strains and found comparable stability. Our initial methods included integration of pRP1195 into RN4220, followed by transduction of the integrated plasmid into the strains NRS384 (USA300), MW2, and Newman. Because phage phi80 can package up to 42 kb of DNA [17], such an approach is less than ideal, as RN4220-specific DNA sequences could potentially be transferred to the target strain. To avoid such a possibility, we subsequently engineered additional luminescent strains by transducing the freely replicating plasmid from RN4220 to the target strains, shifting to the non-permissive temperature for plasmid replication, and isolating integrants. These strains should differ from the parent strains only in the presence of the integrated plasmid and should therefore prove useful in studies of *S. aureus* pathogenesis.
